# miR-183-5p Aggravates Breast Cancer Development via Mediation of RGS2

**DOI:** 10.1155/2021/9664195

**Published:** 2021-11-20

**Authors:** Chihua Wu, Youlin Tuo, Gang Hu, Jing Luo

**Affiliations:** ^1^Department of Breast Surgery, Sichuan Academy of Medical Sciences & Sichuan Provincial People's Hospital, Chengdu 610072, China; ^2^Department of Breast Surgery, Sichuan Provincial People's Hospital, University of Electronic Science and Technology of China, Chengdu 610072, China; ^3^Chinese Academy of Sciences Sichuan Translational Medicine Research Hospital, Chengdu 610072, China

## Abstract

This study mainly explores how miR-183-5p pertains to breast cancer (BC) development. Functional assays were employed to test impacts of miR-183-5p in this cancer. Targeting between RGS2 and miR-183-5p was examined with dual-luciferase assay, and how their interaction pertains to cancer progression was further unraveled. miR-183-5p level was noticeably high in cancer tissue/cells. Overexpressing miR-183-5p could remarkably deteriorate cancer progression. The regulatory gene RGS2 levels was markedly low in BC, and two genes we researched were negatively correlated. It was uncovered by rescue assay that miR-183-5p/RGS2 axis mediated tumor-relevant behaviors in BC. Altogether, miR-183-5p aggravates BC development via mediation of RGS2. miR-183-5p supplies a promising target for BC therapy.

## 1. Introduction

Breast cancer (BC) is a dreaded female disease. In accordance with statistics, 2,090,000 cases were reported all over the world, wherein 627,000 people died from BC in 2018 [1]. High mortality and morbidity of BC can severely influence women's life quality. At present, BC treatment mainly includes surgery, chemotherapy, endocrinotherapy, radiotherapy, and biotherapy [2, 3]. However, the pathogenic process of BC involves a complex effect of multifactor, multistage, and multistep [4], which makes different patients have different reactions to treatment accompanied by a certain strong adverse reaction. In biology, target treatment at molecular level can not only allow us to further tailor therapies for cancer but also avoid developing strong adverse reaction or even reach no side effects [5]. Therefore, it is a current focus of the cancer research field.

MicroRNA (miRNA) is highly evolutionarily conserved and a short noncoding RNA about 22 nucleotides long that promotes mRNA degradation via specifically binding 3′-untranslated region (UTR) of mRNA [6, 7]. miRNAs, a critical part as tumor progresses, regulate target gene to control cell proliferation, differentiation, invasion, and apoptosis, and aberrant miRNA expression is proved to affect BC tumor development and progression [8]. miR-183-5p, involving in cellular processes, is abnormally expressed in a variety of cancers. Studies show that activated miR-183-5p promotes tumor development, including pancreatic, prostate, and non-small-cell lung cancers [9–11]. There remains a shortage of evidence about miR-183-5p in BC, with only a paper finding that miR-183-5p modulates human BC cell proliferation and inhibits cell apoptosis [12].

Hence, questing for the impacts of miR-183-5p in BC retains value. Mechanisms of miR-183-5p on BC cellular processes were sought in the present paper. The present paper raises the prospects of management of BC.

## 2. Materials and Methods

### 2.1. Cell Lines

Normal mammary epithelial cell line MCF-10A and BC cell lines (BT549 and MDA-MB-231) were provided by cell resource center of Institute of Basic Medical Sciences of Chinese Academy of Medical Sciences (resource num. 3111C0001CCC000406, 3111C0001CCC000336, and 3111C0001CCC000014). BC cell lines (MCF-7 and BT474) were offered by the cell bank of China Center for Type Culture Collection (resource num. 3142C0001000001079, 3142C0001000000314). The complete medium used in this study was Roswell Park Memorial Institute (RPMI) 1640 (Gibco, 11875093) containing 10% fetal bovine serum (FBS) (Gibco, 10099141C), and antibiotics were penicillin (100 *μ*g/ml) (Invitrogen, Grand Island, NY, USA) and streptomycin (100 *μ*g/ml) (Invitrogen, Grand Island, NY, USA). All cells were incubated in an incubator under general conditions.

### 2.2. Bioinformatics Analysis

Mature miRNAs, mRNAs, and corresponding clinical data were assessed from The Cancer Genome Atlas- (TCGA-) BRCA of TCGA database, and miR-183-5p expression was analyzed. Differential analysis (logFC | >2.0, *P*adj < 0.01) was undertaken on mRNAs with EdgeR package to obtain differentially expressed genes (DEGs). mRNAs were predicted by TargetScan, miRTarBase, and starBase, and DEGs were intersected with predicted genes to determine the target gene.

### 2.3. Gene Overexpression and Knockdown

miR-183-5p mimics, mimic NC, miR-183-5p inhibitor, and inhibitor NC (GenePharma Company, Shanghai, China) with a concentration of 50 nm were used for transient transfection, respectively. Small interfering RNA (siRNA) targeting RGS2 genes was provided by RiboBio (Guangzhou, China). Recombinant plasmid pEGFP1-RGS2 (oe-RGS2) was constructed by pEGFP1 vector. According to the instruction, Lipofectamine 3000 (Invitrogen, Life Technologies, New York, USA) kit was applied to transfect mimics, inhibitors, siRNAs, recombinant plasmids, and corresponding controls into MDA-MB-231 cells.

### 2.4. Real-Time Fluorescence Quantitative PCR (qRT-PCR)

RNAPure total RNA fast isolation kit (BioTeke, Beijing, China) was used to extract total RNA in cells. To detect miR-183-5p, the specific RT primer (RiboBio, China) was applied for reverse transcription. RNA was reversely transcribed into cDNA with super M-MLV reverse transcriptase (BioTeke). qPCR was undertaken on Roche Light-80 Cycler 480 real-time PCR system (Roche Diagnos-81 tics, Basel, Switzerland). qRT-PCR reaction conditions were as follows: 95°C, 15 min; 35 cycles: 94°C, 15 sec; 55°C, 30 sec; and 72°C, 30 sec. RGS2 and miR-183-5p expressions were normalized with GAPDH and U6 as the internal reference, respectively. Primers used in the experiment are shown in Supplementary Table 1.

### 2.5. Western Blots

Total proteins of MDA-MB-231 cells were extracted, and protein concentration was determined by bicinchoninic acid (BCA) protein assay kit (Beyotime). 15-30 *μ*g protein sample was used for sodium dodecyl sulfate polyacrylamide gel electrophoresis (SDS-PAGE) and then transferred onto a polyvinylidene fluoride membrane (Millipore, Billerica, MA). Thereafter, the membrane was incubated with primary antibodies at 4°C in Tris-buffered saline Tween + 5% skim milk overnight and with secondary antibody for 2 h. Enhanced chemiluminescence (ECL) (7Sea Biotech, Shanghai, China) was used as substrate to detect protein levels. Antibody dilution ratio is shown in Supplementary Table 2. The experiment experienced 3 repetitions.

### 2.6. Cell Proliferation Assay

When MDA-MB-231 cell density reached 80%, the cells were washed with phosphate-buffered saline (PBS) twice. Cells were separated with trypsin. After calculation, cells were inoculated in 96-well plates (3 − 6 × 10^3^ cell/well) with each well containing 200 *μ*l medium, and 6 parallel wells were set. 48 h later, 5 mg/ml MTT solution was added into each well. After 4 h, the medium was removed. OD of each well was measured under 570 nm wavelength with a microplate reader (DNM9606, PuLang, Beijing, China). Cell viability curve was drawn with time as the *x*-axis and OD as the *y*-axis. The experiment was repeated 3 times.

### 2.7. Wound Healing Assay

MDA-MB-231 cells were inoculated in 24-well plates (500 *μ*l each well) with a density of 1 × 10 [6]. After cells were cultured in RPMI 1640 for 16-24 h until cells growing to a monolayer, a 10 *μ*l pipette tip was used to scratch a straight wound on monolayer cells in a 24-well plate. After being washed with PBS 3 times, cells were incubated with fresh medium without FBS for 24 h. Cell migration at 0 h and 24 h was observed with a 100-fold microscope, and photographs were taken.

### 2.8. Transwell Invasion Assay

Cells were inoculated in a Transwell chamber (aperture: 8 *μ*m) at a concentration. Cell suspension was added into the upper chamber with each group 3 parallel chambers. After 24 h, cells on the interior surface of the Transwell chamber were removed with a swab. The lower surface of the Transwell chamber was washed with PBS twice, fixed with 5% formaldehyde, and stained with 0.2% crystal violet staining solution. The crystal violet was eluted with acetic acid solution. Cells were observed and photographed under an invert fluorescence microscope.

### 2.9. Dual-Luciferase Assay

MDA-MB-231 cells were used for dual-luciferase reporter gene assay. MDA-MB-231 cells were inoculated in 12-well plates for 24 h, and then, cells were cultured without serum. After being starved for 1 h, reporter gene plasmids with wild-type (wt) or mutant (mut) RGS2 3′UTR sequences and mimic NC or miR-183-5p mimic were transfected into cells, respectively. Next, cells were cultured generally for 4 h and cultured for another 48 h after changing the medium with complete medium. Luciferase intensity was measured with dual-luciferase reporter system.

### 2.10. Data Analysis

Results were treated adopting SPSS 22.0 statistical software. Measurement data were represented as mean ± SD. *T*-test was utilized to compare two groups. *P* less than 0.05 was significantly statistical. ∗ represents *P* < 0.05.

## 3. Results

### 3.1. Activated miR-183-5p in BC

BC miRNA expression data in TCGA-BRCA were downloaded from TCGA, and miR-183-5p was observed to be conspicuously activated in BC tissue (Figure 1(a)). Moreover, previous results also indicated that miR-183-5p modulates cancer cell proliferation, indicating miR-183-5p an underlying marker [9, 11]. Hence, miR-183-5p was quested here. qRT-PCR method disclosed remarkably higher miR-183-5p levels in BC relative to normal cells (Figure 1(b)). MDA-MB-231 which exhibited the highest miR-183-5p level were subjected to the analyses hereinafter. In all the above, miR-183-5p was markedly activated in BC.

### 3.2. miR-183-5p Aggravates Cellular Processes of BC *In Vitro*

It was exhibited by qRT-PCR that after transfecting miR-183-5p mimic and miR-183-5p inhibitor, MDA-MB-231 cells manifested significantly increased and decreased miR-183-5p, respectively (Figure 2(a)). Furthermore, as examined by cellular functional methods, miR-183-5p mimic markedly accelerated the proliferative (Figure 2(b)), invasive (Figure 2(c)), and migratory (Figure 2(d)) capabilities of BC. Nonetheless, Figures 2(b)–2(d) uncovered the opposite cell capabilities in BC in the miR-183-5p inhibitor group. In all the above, miR-183-5p aggravated cellular processes of BC *in vitro*.

### 3.3. miR-183-5p Constrains RGS2 Levels

2,146 DEGs were acquired from differential expression analysis (1,367 upregulated DEGs and 779 downregulated DEGs) (Figure 3(a)). To increase the reliability of prediction, target genes of miR-183-5p were acquired from prediction based on databases. Four miR-183-5p-mediated differentially expressed mRNAs (DEmRNAs) were gained after the intersection between predicted genes and DEmRNAs (Figure 3(b)). miR-183-5p negatively pertained to RGS2 which was also most relevant to miR-183-5p. Hence, RGS2 was finally chosen for further research (Figures 3(c) and 3(d)). RGS2 was significantly low in BC tissue (Figure 3(e)), and the lower the expression of RGS2 gene, the worse the patient's prognosis (Figure 3(f)). Their binding was predicted via TargetScan (Figure 3(g)). Dual-luciferase method demonstrated hampered luciferase intensity of cells with wt RGS2 3′-UTR carrier upon miR-183-5p overexpression, but no such impacts on cells with mut 3′-UTR carrier (Figure 3(h)). Lastly, qRT-PCR and western blot uncovered the restrained mRNA along with protein levels of RGS2 upon overexpressing miR-183-5p, as opposed to what hampering miR-183-5p triggered (Figures 3(I) and 3(j)). These results represented that miR-183-5p restrained RGS2 levels in BC.

### 3.4. RGS2 Suppresses the Cellular Processes of BC Cells *In Vitro*

RGS2 mRNA levels after overexpressing RGS2 and interfering RGS2 were examined. It was uncovered by qRT-PCR that RGS2 mRNA expression elevated after overexpressing RGS2 while RGS2 mRNA expression significantly declined after silencing RGS2 (Figure 4(a)). Moreover, MTT assay disclosed that overexpressing RGS2 could markedly inhibit BC proliferation, while silencing RGS2 hastened this cell behavior (Figure 4(b)). It was indicated by Transwell assay that overexpressing RGS2 remarkably inhibited BC cell invasive ability while silencing RGS2 markedly promoted BC cell invasive ability (Figure 4(c)). After 24 h of culture after scratching, the wound distance of the oe-RGS2 group was wider than that of NC, while the wound distance in the si-RGS2 group was conspicuously narrowed (*P* < 0.05) (Figure 4(d)). In all the above, RGS2 restrained cell processes of BC *in vitro*.

### 3.5. miR-183-5p Aggravates BC Development by Mediating RGS2

We transfected RGS2 overexpressed vector and miR-183-5p mimics to detect changes of MDA-MB-231 cells in proliferative, invasive, and migratory abilities. It was displayed by qRT-PCR that overexpressing miR-183-5p restrained RGS2 while RGS2 expression was recovered after cotransfecting RGS2 as well (Figure 5(a)). According to MTT assay, overexpressing RGS2 could inhibit miR-183-5p stimulating proliferation of MDA-MB-231 (Figure 5(b)). Transwell and wound healing assays showed that RGS2 could remarkably reverse miR-183-5p accelerating invasive and migratory capabilities of BC (Figures 5(c) and 5(d)). Overall, miR-183-5p targeted RGS2 to accelerate tumor-relevant behaviors in BC.

## 4. Discussion

BC is a lethal tumor among women. Further studies need to be done to eliminate the pain of early death and BC. Compelling evidence disclosed that levels of miRNAs pertain to cancer progression by modulating target protein, which may provide a target for cancer treatment [13, 14]. In relevant studies of cancers, miR-183-5p is a crucial miRNA which can mediate cellular processes in cancers. As earlier papers elaborated, miR-183-5p accelerates tumor differentiation, invasion, and metastasis [15–17] and is critical for cervical cancer, lung cancer, and bladder cancer [18–20]. miR-183-5p can distinguish prostate cancer from benign prostatic hyperplasia [21]. miR-183-5p restrains PTEN to promote lung cancer [11]. However, little is studied about how miR-183-5p influences BC. This study analyzed the miRNA profile of BC and discovered activated miR-183-5p in BC. It was also discovered that miR-183-5p presented markedly high levels in various BC cells, coinciding with bioinformatics outcomes. In the context of previous results, it was speculated that miR-183-5p might stimulate BC progression, which means miR-183-5p is a cancer promoter.

In this article, miR-183-5p was higher in BC than that in normal cells, and overexpressing miR-183-5p notably hastened BC to progress while silencing miR-183-5p caused the opposite result. We predicted the downstream target gene of miR-183-5p as well, and RGS2 was an eligible object to be unraveled. A study confirmed that RGS2 is lowly expressed in BC tissues [22]. RGS2 as a novel regulator of androgen receptor signaling inhibits the development of prostate tumor [23]. Moreover, it was also proved that miR-183-5p could mediate RGS2. Overexpressing RGS2 constrained cell functions in BC while knocking down RGS2 accelerated BC cell progression. After simultaneously overexpressing miR-183-5p and RGS2, it was displayed that RGS2 could partly control miR-183-5p mediating cell functions of BC. Overall, miR-183-5p can deteriorate the progression of BC by RGS2 modulation. Nevertheless, in-depth experiments using cells like MCF-10A were required to examine whether miR-183-5p/RGS2 axis affects BC.

All in all, it was found in this study that activated miR-183-5p in BC can hasten proliferative, invasive, and migratory capabilities of BC cells. A further mechanism is that miR-183-5p aggravated BC via mediation of RGS2. The results enable us a clearer acquisition of miR-183-5p in BC and provide theoretical bases for finding new target therapies of BC.

## Figures and Tables

**Figure 1:** miR-183-5p is activated in BC: (a) boxplot of miR-183-5p expression in the normal group and tumor group; (b) different expressions of miR-183-5p in breast cancer cells shown by qRT-PCR. ∗ represents *P* < 0.05.

**Figure 2:** miR-183-5p deteriorates cellular processes in BC: (a) miR-183-5p expression in BC cells upon overexpressing or silencing miR-183-5p; (b) changes of cell proliferative ability of BC; (c) invasive ability of BC cells (×100); (d) changes of cancer cell migratory capabilities (×40). ∗ represents *P* < 0.05.

**Figure 3:** miR-183-5p restrains RGS2 level: (a) volcano plot of DEmRNAs; (b) overlap between predicted targets and differentially downregulated mRNAs; (c) Pearson correlation between miR-183-5p and predicted targets; (d) correlation between two researched objects in BC; (e) boxplot of RGS2 expression; (f) survival analysis of RGS2 genes; (g) predicted binding sites between two researched objects; (h) the luciferase intensity measured; (i) changes of RGS2 mRNA expression after overexpressing and silencing miR-183-5p; (j) RGS2 protein expression in BC. ∗ represents *P* < 0.05.

**Figure 4:** RGS2 suppresses cellular behaviors of BC *in vitro*: (a) the expression of RGS2 in BC cells after overexpressing/interfering RGS2; (b) BC cell proliferative ability after overexpressing/interfering RGS2; (c) BC cell invasive ability after overexpressing/interfering RGS2 (×100); (d) results of wound healing assay of BC (×40). ∗ represents *P* < 0.05.

**Figure 5:** Rescue assay verifies that miR-183-5p downregulates RGS2 to accelerate cell functions in BC: (a) changes in mRNA level of RGS2 after cotransfecting miR-183-5p and RGS2; (b) effects of simultaneously overexpressing miR-183-5p and RGS2 on BC cell activity; (c) effects of simultaneously overexpressing miR-183-5p and RGS2 on the invasive ability of BC (×100); (d) changes of wound healing areas in BC in each group after simultaneously overexpressing miR-183-5p and RGS2 (×40). ∗ represents *P* < 0.05.

## Data Availability

The data and materials in the current study are available from the corresponding author on reasonable request.

## Supplementary Materials

Supplementary 1 Supplementary Table 1: primer sequence list used in qRT-PCR.

Supplementary 2 Supplementary Table 2: antibody information used in western blot in the laboratory.
